This article has been retracted.

# Single-Cell Transcriptional Profiling Reveals Low-Level Tragus Stimulation Improves Sepsis-Induced Myocardial Dysfunction by Promoting M2 Macrophage Polarization

**DOI:** 10.1155/2022/3327583

**Published:** 2022-10-15

**Authors:** Yufan Yang, Longlong Xie, Yinghui Peng, Haipeng Yan, Jiaotian Huang, Zhenghui Xiao, Xiulan Lu

**Affiliations:** ^1^Department of Pediatric Intensive Care Unit of Hunan Children's Hospital, No. 86 Ziyuan Road, Changsha, Hunan 410007, China; ^2^Pediatrics Research Institute of Hunan Province, Hunan Children's Hospital, No. 86 Ziyuan Road, Changsha, Hunan 410007, China; ^3^Department of Ultrasound of Hunan Children's Hospital, No. 86 Ziyuan Road, Changsha, Hunan 410007, China

## Abstract

**Background:**

Sepsis can lead to multiple organ damage, of which the heart is one of the most vulnerable organs. Vagal nerve stimulation can reduce myocardial injury in sepsis and improve survival rates. However, the potential impact of low-level tragus stimulation and disparate cell populations on sepsis-induced myocardial dysfunction remains undetermined.

**Methods:**

A cardiac single-cell transcriptomic approach was used for characterizing cardiac cell populations that form the heart. Single-cell mRNA sequencing data were used for selecting all cardiac macrophages from CD45^+^ cells. Then, echocardiography, western blot, flow cytometry, immunofluorescence, and immunohistochemistry were performed to verify the single-cell mRNA sequencing results.

**Results:**

Using single-cell mRNA sequencing data, we uncovered the multiple cell populations contributing to myocardial injury in sepsis under low-level tragus stimulation, thereby illustrating a comprehensive map of the cardiac cellular landscape. Pseudotiming analysis in single-cell sequencing showed that low-level vagal nerve stimulation played an anti-inflammatory role by promoting cardiac monocytes into M2 macrophages, which significantly increased *α*7nAChR expression in heart tissues. Echocardiography assessment indicated that low-level vagal nerve stimulation could also improve cardiac functions in mice with sepsis-induced myocardial dysfunction. In addition, the heart tissues of mice from the sepsis group with low-level tragus stimulation had significantly lower interleukin-1*β* expression levels than those from the sepsis group. Flow cytometry analysis showed that different acetylcholine concentrations promoted cardiac monocytes into M2 macrophages in *in vitro* experiments.

**Conclusion:**

Low-level tragus stimulation could improve sepsis-induced myocardial dysfunction by promoting cardiac monocytes to M2 macrophages.

## 1. Introduction

Sepsis can lead to multiple organ dysfunction, of which the heart is one of the most vulnerable organs that could be affected [1]. Recent studies showed that inflammation is the main cause of myocardial injury in sepsis [2], leading researchers to actively investigate strategies that could effectively inhibit sepsis-induced inflammation in the septic heart to reduce myocardial injury and improve cardiac functions. In this regard, it was reported that vagal nerve stimulation could reduce sepsis-induced myocardial injury and improve survival rates [3]. However, due to its invasive approach, the application of implanted vagal nerve stimulation has been limited [4]. The auricular branch of the vagus nerve is the only superficially distributed afferent vagus nerve close to the skin surface [5]. A previous report showed that low-level tragus stimulation (LL-TS) could promote blood flow and reduce reperfusion injury in patients with myocardial infarction [6]. However, there is no literature on whether LL-TS could be used to prevent and treat myocardial dysfunction in sepsis. Thus, considering that conventional vagal nerve stimulation may reduce heart rate and blood pressure, we propose using a low-level transcutaneous electrical stimulation to the auricular vagal nerve as an approach for noninvasive vagal nerve stimulation.

Single-cell mRNA sequencing was shown to effectively characterize macrophage heterogeneities in heart diseases [7, 8]. In addition, the use of several dimension reduction methods, clustering models, and comparative analyses of single-cell RNA sequencing data provides further insights into cellular heterogeneity and deepens our understanding of individual cell functions [9]. Studies have shown that polarization of cardiac M2 macrophages can improve left ventricular function after myocardial infarction [10]. However, the relationship between M2 macrophage polarization and sepsis-induced cardiac dysfunction has not been explored.

This study was performed to identify macrophages associated with cardiac dysfunction, investigate their roles in sepsis-induced myocardial dysfunction, and determine the efficacy of LL-TS in improving cardiac functions during sepsis. Altogether, our results showed that low-level tragus stimulation could improve sepsis-induced myocardial dysfunction by promoting cardiac monocytes to M2 macrophages.

## 2. Methods

### 2.1. Animal Models

Specific pathogen-free (SPF) 6- to 8-week-old C57BL male mice weighing 20-25 g were obtained from the animal experiment center of Hunan Children's Hospital. The mice were kept under the experimental condition for at least one week. Before cecal ligation and puncture operation (CLP), solid and liquid fasting was performed to ensure the consistency of intestinal conditions. Isoflurane inhalation anesthesia was used, after which the abdominal body hair of the mice was removed, and they were conventionally sterilized. The mice were covered with a sterile towel, and a 1 cm incision was made along the midline of their abdomen. The cecum was identified, and the blind end was carefully dissociated to avoid vascular injury. Then, the cecum was sutured at the far side of the ileocecal valve and 1 cm from the end of the cecum. Care was taken to avoid ligating the mesenteric vessels of the ileum and cecum. The no. 7 needle was used to penetrate the cecum once, some intestinal content was squeezed out, the cecum was then carefully placed back into the abdominal cavity, and each layer of the abdominal wall was sutured to close the incision. After the operation, 30 mL/kg of normal saline was injected intraperitoneally for fluid resuscitation, and the animals were put back into their respective feeding cage. After waking from the anesthesia, the mice could move, eat, and drink water [11]. The mice were divided into the following four groups: control, sham, CLP, and CLP+LL-TS groups, with five mice per group.

### 2.2. Low-Level Tragus Stimulation

Auricular vagal nerve stimulation (tragus stimulation) was performed as previously reported [12]. Briefly, using a 20 Hz frequency and 1 ms pulse width, bilateral tragus stimulation was given via a duty cycle of 5 s on and 5 s off delivered to the external auditory canal via ear clips attached to a custom-made stimulator. The voltage was then gradually increased until the sinus rate of the mice was slowed, which was then used as the threshold voltage based on which LL-TS was given at 80% below the threshold voltage [5]. The delivered electric voltage ranged between 0.3 and 1 mV, did not change the heart rate of the mice, and had no serious adverse reactions that could relate to an increase in plasma epinephrine level. LL-TS was given 30 minutes every day for 3 weeks, following which CLP operation for the sepsis model was performed.

### 2.3. Single-Cell mRNA Sequencing

The mice's heart was cut into two pieces, one of which was enzymatically digested, while the other was also digested and immune cells were sorted by CD45 magnetic beads. CD45-sorted positive cells were mixed with nonsorted cells after enzymatic digestion of the same tissue block in a 1 : 1 proportion. The 10x Genomics GemCode technology was used to encapsulate the single cells in droplets, which were then processed by OE Biotech. Co., Ltd. (Shanghai, China). A unique molecular identifier (UMI) was used to barcode every cell and transcript, and a Single-Cell 30 Reagent Kit v2 (10X Genomics) was used to generate cDNA for sequencing on the Illumina platform. The libraries were sequenced on the HiSeq 2500 platform with paired-end sequencing. The raw sequencing data were uploaded to GSE207363.

### 2.4. Sequencing Analysis

Demultiplexing, quantification, and filtering of the data were performed using CellRanger (version 5.0.0). The mice's UCSC mm10 reference genome was used to align the reads, which were then used to quantify the expression levels of the mice's genes and generate a gene-barcode matrix. Uniform Manifold Approximation and Projection (UMAP) clustering and comparison were performed using Seurat version 3.1.2 and Monocle 2 version 2.4.0. The cell types of single cells were annotated with the SingleR package (version 0.2.2) and two mouse databases (ImmGenData and MouseRNAseqData). The AddModuleScore function in Seurat was used with default settings. We used 4 well-defined gene markers (Adgre1, Itgam, Fcgr1, and Cd68) to define macrophages and 4 well-defined gene markers (Lyz2, Ly6c2, Plac8, and Cd14) to define monocyte [13].

### 2.5. Mouse Echocardiography

Philips EPIQ7C (Philips Ultrasound, Inc., Bothell, USA) was used for echocardiography under isoflurane anesthesia, as described above. The left ventricular ejection fraction (EF) and fractional shortening were estimated using the end-diastole and end-systole left ventricular internal diameters, measured vertically on the long axis of the ventricle.

### 2.6. Immunofluorescence and Immunohistochemical Analyses

The mouse hearts were fixed in formalin supplemented with 30 mM KCl (Sigma Aldrich), paraffin-embedded (FFPE), and then sectioned at 10 *μ*m thickness for immunofluorescence and immunohistochemical staining. For fluorescence imaging, the sections were stained with antibodies targeting F4/80 (F4/80; 1 : 200, sc-71085, Santa Cruz Biotechnology) and *α*7 nicotinic acetylcholine receptor (*α*7nAChR) (*α*7nAChR; 1 : 200, ab216485, Abcam) and additionally stained using DAPI (1 *μ*g/mL, D9542, Sigma Aldrich) before acquiring confocal micrographs. Micrographs were processed with the Imaris software (Bitplane). For immunohistochemical staining, the heart sections and tragus tissues were stained with antibodies targeting choline acetyltransferase (ChAT) (ChAT; 1 : 200, ab178850, Abcam).

### 2.7. Western Blotting

The heart of mice from each group was used for western blotting. Briefly, they were homogenized using a radioimmunoprecipitation lysis buffer (Sigma, St Louis, USA) containing a proteinase inhibitor (Solarbio, Beijing, China) and centrifuged for 10 min at 4°C. The supernatant was further centrifuged for 20 min. A protein assay kit (Thermo Fisher, Waltham, USA) was then used to assess the protein concentration of each supernatant. Samples with equal amounts of protein were separated using 15% sodium dodecyl sulfate-polyacrylamide gel electrophoresis gel (Bio-Rad). They were then transferred onto an Immobilon membrane (Millipore, Billerica, MA), and after blocking with BlockAce (Dainippon Pharmaceutical, Japan), primary antibodies, including polyclonal antibody for *α*7 nicotinic acetylcholine receptor (*α*7nAchR, Abcam, Cambridge, England), and *β*-actin (internal control, Cell signal Technology) were used at the recommended concentration based on the manufacturer's instructions and dilution ratio of 1 : 3000. The proteins were then detected using enhanced chemiluminescence (Invitrogen). The bands were analyzed on the ECL detection system (GE Healthcare). All experiments were performed in triplicate and repeated at least three times. The quantitative analysis was the ratio of the target protein and *β*-actin for western blot.

### 2.8. Flow Cytometry

Here, we verified whether acetylcholine could stimulate the differentiation of monocytes to the M2 phenotype. Different acetylcholine concentrations (0.5 *μ*g/mL, 1 *μ*g/mL, 2 *μ*g/mL, and 4 *μ*g/mL) of human myeloid leukemia mononuclear cells (THP-1), which is the monocytic cell line, were used to stimulate THP-1 for 24 hours. Then, the cells were washed with phosphate-buffered saline (PBS) containing 1% FBS and 1% Hepes and stained using CD11b (5 *μ*g/mL, Biolegend), CD206 (5 *μ*g/mL, Biolegend), and CD86 (1 *μ*g/mL, Biolegend) antibodies for 30 min at room temperature. THP-1 cells were cultured in RPMI-1640 (Gibco, USA) supplemented with 10% FBS (BI, Israel) and penicillin/streptomycin in a humidified incubator at 37°C and 5% CO_2_. The data were collected using LSRFortessa™ FACS (BD Bioscience) and analyzed using FlowJo software.

### 2.9. Data Analysis

Statistical analyses were performed using SPSS version 18.0 (IBM, Armonk, NY, USA) and GraphPad Prism 8 for Mac (GraphPad Software Inc., La Jolla, CA). The Kruskal-Wallis test was used to determine the significance between group comparisons, and Dunn's multiple comparison test was performed for post hoc pairwise comparisons. *P* < 0.05 was used as the threshold to demarcate statistical significance.

## 3. Results

### 3.1. Effects of Low-Level Tragus Stimulation on Left Ventricular Function

Our results showed comparable echocardiographic baseline measurements between the four mouse groups (Figure 1). Further, 12 hours after cecal ligation and puncture operation, we found that the sepsis group had significantly lower LVEF and LVFS than the control and sham groups (*P* < 0.05). However, treatment with LL-TS significantly improved the LVEF and LVFS of mice compared with the sepsis group (*P* < 0.05).

### 3.2. Single-Cell mRNA Sequencing Data

According to the protocol, we performed single-cell mRNA sequencing 24 hours after CLP operation for the sepsis model. A total of 11 major cell types, comprising macrophages, B cells, cardiomyocytes, dendritic cells (DC), endothelial cells, fibroblasts, granulocytes, pericytes, Schwann cells, smooth muscle cells, and T-natural killer (T-NK) cells, were identified based on the canonical gene marker expressions (Figure 2(a)).

CD45^+^ cell screening and sequencing quality control filters were performed in the four control groups, and dimensionality reduction clustering and enrichment analysis were performed for cardiac macrophages. After applying quality control filters, 3978, 3101, 1850, and 3512 macrophages from the control, sham, sepsis, and sepsis with LL-TS groups were included in the single-cell mRNA sequencing analysis, respectively (Figure 2(b)). The results showed that the macrophage clusters of the sepsis group significantly differed from those of the sepsis with LL-TS group (Figure 2(b)). The sepsis group mainly contained subsets 4 and 9, while the sepsis with LL-TS group mainly contained subsets 3 and 7 (Figures 2(c) and 2(d)). The distribution of M2 macrophages labeled with Mrc1/Cd206 and Cd163 in the sepsis with LL-TS group (subset 3 and subset 7) was higher than that in the sepsis group (subset 4 and subset 9), indicating that LL-TS in sepsis could promote the polarization of cardiac M2 macrophages and inhibit cardiac inflammation (Figure 3).

Pseudotime analysis was performed in the macrophage and monocyte subsets of the sepsis group and the sepsis with LL-TS group. The macrophage and monocyte subsets superimposed on the pseudotime trajectory produced by the Monocle package revealed that monocytes differentiated into M2 macrophages in the sepsis with LL-TS group (Figures 4(k) and 4(l)), while in the sepsis group, the number of M2 macrophages decreased over time (Figures 4(h) and 4(i)). An increasing trend in CD163 and Mrc1 mRNA levels in the sepsis with LL-TS group was observed (Figures 5(e) and 5(f)), while that of the sepsis group exhibited a decreasing trend (Figures 5(g) and 5(h)).

### 3.3. LL-TS Reduced Cardiac Inflammation in Septic Mice

We observed a significantly higher expression level of IL-1*β* in the heart tissues of the septic mice than in the sham and control groups (*P* < 0.05) (Figure 6) and a significantly lower IL-1*β* expression level in the sepsis with LL-TS group than in the sepsis group (*P* < 0.05) (Figure 6). These findings indicated that LL-TS could significantly reduce cardiac inflammation in septic mice.

### 3.4. LL-TS Increased Cardiac *α*7nAChR Expression and Macrophages

Further, immunofluorescence experiments showed that LL-TS significantly increased *α*7nAChR expression in the mice's heart (Figure 7) and macrophages (Figure 8), indicating that LL-TS might improve sepsis-induced cardiac dysfunction by activating the cardiac cholinergic anti-inflammatory pathway.

### 3.5. LL-TS Increased the Secretion of Cardiac Acetylcholine

After LL-TS, the immunohistochemistry of the heart and auricula showed positive acetylcholinesterase staining, indicating the secretion of acetylcholine at the end of the vagal nerve in the heart was increased (Figures 9 and 10) and the presence of vagal nerve distribution in the stimulating tragus area.

### 3.6. Acetylcholine Can Promote THP-1 into the Phenotype of M2 Macrophage

Further experiments using 0.5 *μ*g/mL, 1 *μ*g/mL, 2 *μ*g/mL, and 4 *μ*g/mL of acetylcholine to stimulate THP-1 for 24 hours showed that different concentrations of acetylcholine stimulated THP-1 into M2 macrophages (Supplementary Figure 1) (Figure 11).

## 4. Discussion

In this study, we investigated the effects of LL-TS on sepsis-induced cardiac dysfunction using single-cell sequencing. The results showed that intermittent LL-TS treatment could significantly improve cardiac functions and reduce heart inflammation by promoting cardiac M2 macrophage polarization in septic mice and that these processes might be related to the activation of the cholinergic anti-inflammatory pathway.

### 4.1. LL-TS Reduced Cardiac Inflammation in Septic Mice

It was confirmed that vagal nerve stimulation improved systemic inflammatory responses and survival rates of CLP sepsis model animals [14]. Stavrakis et al. recently reported that postoperative atrial fibrillation and inflammation could be suppressed by low-level vagal nerve stimulation [15]. In this present study, we observed reduced cardiac inflammation after the CLP operation following LL-TS treatment based on the decreased expression level of protein IL-1*β* in the heart tissues of septic mice.

### 4.2. Improvement of Sepsis-Induced Cardiac Dysfunction following LL-TS Treatment

We also showed that LL-TS treatment and chronic intermittent LL-TS treatment by enhancing vagal nerve activity alleviated sepsis-induced cardiac dysfunction based on increased LVEF and LVFS. Similar findings were also reported by Zhou et al. [16] using chronic intermittent LL-TS in a rat model of heart failure with preserved ejection fraction (HFpEF), indicating the promising potential clinical applicability of LL-TS as a noninvasive neuromodulation therapy for HFpEF.

### 4.3. LL-TS Promoted the Cardiac M2 Macrophage Polarization

An increase in inflammation during sepsis is often caused by the release of cytokines after the activation of innate immune cells such as macrophages. Inflammation is the main factor inducing myocardial injury and dysfunction. Studies have shown that macrophages comprised M1 and M2 phenotypes [17]. M1 macrophages can secrete proinflammatory cytokines that have proinflammation roles, while M2 macrophages release anti-inflammatory cytokines that play anti-inflammation roles. Macrophage polarization balance is key for effective toxin removal and tissue repair, and regulating macrophage polarization is of great significance in improving sepsis-induced cardiac dysfunction. The activation of *α*7nAChR was shown to inhibit M1 microglia transformation and promote the M2 phenotype, leading to changes in vagal nerve neuroinflammation in various diseases of the central nervous system [18]. Although several studies have reported that *α*7nAChR activation promoted M2 macrophage polarization [19–21], no research has investigated the effects of LL-TS on the phenotypic transformation of macrophages in sepsis-induced cardiac dysfunction. In this study, we found that LL-TS treatments increased *α*7nAChR expression. Also, through CD45^+^ cell screening and sequencing quality control, we observed that LL-TS induced the polarization of M2 macrophages.

### 4.4. Possible Mechanisms of LL-TS on Vagal Nerve

The vagal nerve's auricular branch innervates the auricular concha and most of the auditory meatus [22] and terminates mainly in the nucleus of the solitary tract [23], where many autonomic nerve fibers, including those in the heart, often project [24, 25]. Gao et al. [26] discovered that acupuncture-like stimulation of the vagal nerve's auricular branch had inhibitory effects on the cardiovascular system due to activation of cardiac-related neurons in the nucleus of the solitary tract. Wang et al. [5] found that LL-TS had similar effects as invasive cervical vagal nerve stimulation on the vagal efferent fibers, which are part of the final pathway responsible for the regulation of the intrinsic cardiac autonomic nervous system. Thus, cardioprotective effects can be achieved via electric stimulation of the vagal nerve's auricular branch due to increased vagal tone from afferent vagal nerve activation and modulation of the intrinsic cardiac autonomic nervous system.

### 4.5. Study Limitations

First, no *in vivo* validation studies were performed to confirm whether acetylcholine promoted monocyte transformation into M2 macrophages due to the small number of monocytes in the heart of the mouse models. Second, we did not detect the vagal nerve activity value, which might have revealed the relationship between vagal nerve activity and LL-TS. Third, the study design did not include blood pressure measurements of the mice, which could be an important indicator. Thus, additional investigations are needed to confirm our findings.

## 5. Conclusion

Low-level tragus stimulation might improve sepsis-induced myocardial dysfunction by promoting cardiac monocytes to M2 macrophages.

## Figures and Tables

**Figure 1:** Echocardiography of mice in each group. (a) Control group. (b) Sham group. (c) Sepsis group. (d) Sepsis+LL-TS group. (e) Comparison of left ventricular ejection fraction (LVEF) value among the 4 groups; ^∗^*P* < 0.01 sepsis group vs. sham group, ^∗∗^*P* < 0.01 sepsis group vs. sepsis+LL-TS group. (f) Comparison of left ventricular fractional shortening (LVFS) value among the four groups; ^#^*P* < 0.01 sepsis group vs. sepsis+LL-TS group, ^##^*P* < 0.01 sepsis group vs. sepsis+LL-TS group. LVEF: left ventricular ejection fraction; LVFS: left ventricular fractional shortening; LVDd: left ventricular end-diastolic dimension; LVDs: left ventricular end-systolic dimension.

**Figure 2:** Dimension reduction cluster analysis and enrichment analysis for cardiac macrophages. (a) Major cardiac cell populations identified after unsupervised clustering. Each point depicts a cell cluster, colored according to cluster designation. (b) Dimension reduction cluster analysis of macrophages in control, sham, sepsis, and sepsis with LL-TS groups. (c) UMAP image of cardiac macrophage subset clusters. (d) Cardiac macrophage subset cluster in each group.

**Figure 3:** The Mrc1 and Cd163 mRNA expression in each group. (a) The UMAP diagram of Mrc1 mRNA expression of macrophages in the sepsis group. (b) The UMAP diagram of Cd163 mRNA expression of macrophages in the sepsis with LL-TS group. (c) The violin diagram of Mrc1 mRNA expression in macrophage subset clusters. (d) The violin diagram of Cd163 mRNA expression in macrophage subset clusters. (e) The significant differences of Mrc1 mRNA expression between the sepsis and sepsis with LL-TS groups. (f) The significant differences of Cd163 mRNA expression between the sepsis and sepsis with LL-TS groups. This figure indicates that LL-TS inhibits cardiac inflammation by promoting M2 macrophage polarization.

**Figure 4:** The pseudotime analysis of macrophages in each group. (a) Pseudotime trajectory of monocytes and macrophages in the control group. (b) Pseudotemporal analysis of Mrc1^+^ macrophages (M2 macrophages) differentiation in the control group. (c) Pseudotime sequence analysis of monocyte and macrophage differentiation in the control group. (d) Pseudotime trajectory of monocytes and macrophages in the sham group. (e) Pseudotemporal analysis of Mrc1^+^ macrophage (M2 macrophage) differentiation in the sham group. (f) Pseudotime sequence analysis of monocyte and macrophage differentiation in the sham group. (g) Pseudotime trajectory of monocytes and macrophages in the sepsis group. (h) Pseudotemporal analysis of Mrc1^+^ macrophage (M2 macrophage) differentiation in the sepsis group. (i) Pseudotime sequence analysis of monocyte and macrophage differentiation in the sepsis group. (j) Pseudotime trajectory of monocytes and macrophages in the sepsis with LL-TS group. (k) Pseudotemporal analysis of Mrc1^+^ macrophage (M2 macrophage) differentiation in the sepsis with LL-TS group. (l) Pseudotime sequence analysis of monocyte and macrophage differentiation in the sepsis with LL-TS group. This figure indicates that LL-TS promotes the differentiation of monocytes to M2 macrophages.

**Figure 5:** The Mrc1 and Cd163 expression of each individual cell in each group, from monocyte differentiation to macrophages. (a) The Mrc1 expression of each individual cell in the control group. (b) The CD163 expression of each individual cell in the control group. (c) The Mrc1 expression of each individual cell in the sham group. (d) The CD163 expression of each individual cell in the sham group. (e) The Mrc1 expression of each individual cell in the sepsis group. (f) The CD163 expression of each individual cell in the sepsis group. (g) The Mrc1 expression of each individual cell in the sepsis with LL-TS group. (h) The CD163 expression of each individual cell in the sepsis with LL-TS group. As is shown in the figure, Mrc1 and CD163 mRNA expression increased significantly from monocyte differentiation to macrophages in the sepsis with LL-TS group. However, in the sepsis group, Mrc1 and CD163 mRNA expression increased at first and then decreased as time goes on.

**Figure 6:** Protein IL-1*β* expression levels of mouse heart in each group. (a) The representative figure of protein IL-1*β* expression levels of mouse heart in each group. (b) Comparison of protein IL-1*β* relative expression levels of heart tissue of each group. ^∗^*P* < 0.01 sepsis group vs. sepsis with LL-TS group, ^∗∗^*P* < 0.01 sepsis group vs. sepsis with LL-TS group. This figure demonstrates that the protein IL-1*β* expression in heart tissue in the sepsis with LL-TS group significantly decreases comparing with the sepsis group, indicating that LL-TS reduces the cardiac inflammation in septic mice.

**Figure 7:** Protein *α*7nAChR expression levels of mouse heart in each group. (a) The representative figure of protein *α*7nAChR expression levels of mouse heart in each group. (b) Comparison of protein *α*7nAChR relative expression levels of heart tissue of each group. ^∗^*P* < 0.01 sepsis group vs. sepsis with LL-TS group. This figure demonstrates that the protein *α*7nAChR expression in heart tissue in the sepsis with LL-TS group significantly increases, indicating that LL-TS activates the cardiac cholinergic anti-inflammatory pathway.

**Figure 8:** The immunofluorescence staining of *α*7nAChR and F4/80 in each group. This figure demonstrates that LL-TS can significantly increase the *α*7nAChR expression on cardiac macrophages, indicating that LL-TS can improve sepsis-induced myocardial dysfunction by activating cardiac cholinergic anti-inflammatory pathway and regulating macrophages.

**Figure 9:** The expression of ChAT of mouse heart in each group detected by immunohistochemistry. (a) Control group. (b) Sham group. (c) Sepsis group. (d) Sepsis with LL-TS group. The red arrow in (d) indicates that ChAT is positive. This figure demonstrates that LL-TS can increase the secretion of ChAT, indicating that LL-TS can increase the secretion of acetylcholine from the ending of vagal nerve. Also, it indicates that the LL-TS is effective.

**Figure 10:** The expression of ChAT of mouse heart in each group detected by immunohistochemistry. (a) Control group. (b) Sham group. (c) Sepsis group. (d) Sepsis with LL-TS group. The black arrows in (a)–(c) show nerve distribution, and the immunohistochemistry of ChAT is negative. The red arrow in (d) indicates the nerve distribution, and the immunohistochemistry of ChAT is positive. This figure demonstrates that the vagal nerve is distributed on the tragus of mice. And it demonstrates that LL-TS can increase the secretion ChAT of vagal nerve on the tragus of mice, indicating that LL-TS can increase the secretion of acetylcholine from the ending of vagal nerve.

**Figure 11:** Different concentrations of acetylcholine to stimulate THP-1. (a) The mean fluorescence intensity of CD206 increased significantly in different concentrations of acetylcholine compared with the control group. (b) The difference between the groups was statistically significant.

## Data Availability

The data that support the findings of this study are available from the first author Yufan Yang, upon reasonable request.

## Supplementary Materials

Supplementary Materials Supplementary Figure 1: the FACS gating strategy. Firstly, we selected the CD11b-positive macrophage. And then, we selected the CD86-negative macrophage. And we used the FlowJo software to analyze the change of CD206 phenotype in the end.
